The article "Construction of AI Environmental Music Education Application Model Based on Deep Learning" was retracted in 2023. Reasons: unreliable results or conclusions; concerns about the data; concerns about the results or conclusions; concerns about the peer review.

# Construction of AI Environmental Music Education Application Model Based on Deep Learning

**DOI:** 10.1155/2022/6440464

**Published:** 2022-08-22

**Authors:** Chaozhi Cheng, Yujun Xiao

**Affiliations:** Huaihua University, Huaihua 418000, China

## Abstract

The art of music, which is a necessary component of daily life and an ideology older than language, reflects the emotions of human reality. Many new elements have been introduced into music as a result of the quick development of technology, gradually altering how people create, perform, and enjoy music. It is incredible to see how actively AI has been used in music applications and music education over the past few years and how significantly it has advanced. AI technology can efficiently pull in the course, stratify complex large-scale music or sections, simplify teaching, improve student understanding of music, solve challenging student problems in class, and simplify the tasks of teachers. The traditional music education model has been modified, and the music education model's audacious innovation has been made possible by reducing the distance between the teacher and the student. A classification algorithm based on spectrogram and NNS is proposed in light of the advantages in image processing. The abstract features on the spectrogram are automatically extracted using the NNS, which completes the end-to-end learning and avoids the tediousness and inaccuracy of manual feature extraction. This study, which uses experimental analysis to support its findings, demonstrates that different music teaching genres can be accurately classified at a rate of over 90%, which has a positive impact on recognition.

## 1. Introduction

The use of AI technology, a new technical science, to simulate, develop, expand, and extend human intelligence is now possible thanks to the rapid advancement of science and technology. It combines many academic fields, such as computer science, psychology, philosophy, and many others, to create interdisciplinary knowledge that can be applied to all facets of daily life. AI technology has been combined and developed with music education today as a result of the quick development of music education, and it has now emerged as the next big thing in music education. It is important not to undervalue the monumental advancement in education. The traditional teaching concept and mode have been greatly impacted by this new teaching approach, which has also created a development path that is diversified, multi-level, and situational. For the combined development of the teaching field and information technology development, it has emerged as a new trend and direction. Additionally, significant changes have been made to the way that music is taught [1]. Students can use this new musical system to perceive music and enjoy the beauty of each note, but they can also use this artificial intelligence (AI) program regardless of the musical concepts that teachers teach in the classroom. By actually playing, students are better able to comprehend the music theory that their teacher has taught them as well as the qualities and purposes of each musical element. The teacher can play a question in music class, then the students can play another response, or the teacher can play a piece of music, and then the students can repeat it or recreate it [2, 3]. Both music students and music teachers benefit from the convenience that AI technology and music software combine to offer.

Only regular classrooms and school music classrooms use the traditional educational model. The instructional design is straightforward. The majority of music educators impart theoretical knowledge, and in order to learn, students mimic their ideas and rhythms. The teaching format is fairly straightforward. In addition, students' lack of interest in learning music results in low classroom learning efficiency, which is detrimental to the promotion and advancement of music. This is because many objective factors, such as time and space, have an influence on and limitations on learning. The ease of the Internet, mobile Internet, and other new models have recently given education a new learning environment with the arrival of the information network era. By removing the arbitrary limitations of time and location, the network era has expanded the time and space of music education. To meet the various learning needs of students at various stages, there is still insufficient personalization. This not only enhances the musical experience for students, but it also fosters interaction and communication between them and their teachers. Students will transition from being passive to being active in the classroom in this way. Instead of just listening to the teacher explaining things, they can now actually experience and comprehend music thanks to the AI system. On this system, they are able to feel the music that the teacher cannot study and comprehend [4]. Students can better understand the traits and purposes of each musical element through the use of this AI software, as well as how these musical elements are created during the creation process. The network era's approach to music education has been further enhanced with the arrival of the AI era, and it is now moving toward in-depth socialization. In addition to completing fundamental teaching tasks, advanced AI can also enhance different postclass phases to better serve students. Education penetrates society deeper by meeting the various musical needs of students at various stages of their education.

Artificial intelligence (AI) technology can quickly stratify complex, large-scale music or sections, simplify instruction, improve student understanding of music, efficiently solve students' challenging class problems, make tasks for teachers simpler, and successfully pull in the course. The bold innovation of the music education model has been realized, the distance between the teacher and the student has been reduced, and the conventional music education model has been modified. This paper suggests a classification algorithm based on spectrogram and NNS [5] based on the benefits of deep learning in image processing. The end-to-end learning is finished by using the NNS to automatically extract the abstract features on the spectrogram in order to avoid the tediousness and imprecision of manual feature extraction. This study examines how two different NNS structures affect the classification of musical genres. The long-term memory network created in this paper to classify music genres uses the manually extracted time series features of music as training data [6]. The impact of various characteristics on the classification of musical genres is investigated through comparative experiments.

The originality of this paper is as follows: genre classification in music education is a significant area of music information retrieval. To increase the effectiveness of music instruction, accurate music classification is crucial. Artificial intelligence (AI) technology can quickly stratify complex, large-scale music or sections, simplify instruction, improve student understanding of music, efficiently solve students' challenging class problems, make tasks for teachers simpler, and successfully pull in the course. The bold innovation of the music education model has been realized, the distance between the teacher and the student has been reduced, and the conventional music education model has been modified. This study uses NNS to categorize the various types of music instruction and uses experiments to examine the benefits and drawbacks of various models.

## 2. Related Work

Humans first developed the new theory of artificial intelligence in the 1950s, along with related technology. McCarthy had first put forth the idea as a novel one. AI has been extensively utilized in every aspect of human life as a new tool and technology. Machine learning research is incorporated into the burgeoning field of deep learning. His goal is to create a NNS that can mimic the human brain's mechanism for data analysis by first simulating the human brain's ability to learn and analyze information and then building a human brain from scratch. Its primary characteristic is an attempt to mimic the way that the neurons in the brain transmit and process information, just like its predecessor, the artificial NNS. As science and technology have advanced quickly, more effective, considerate, and intelligent synthesizers have been adopted by the music teaching market and classrooms [7, 8].

Chen et al. conducted in-depth research on MIDI when studying music classification algorithms based on deep learning models and extracted 100 features from musical information such as musical instruments, composition, rhythm, pitch, melody, and chords, using machine learning classifiers such as the nearest neighbor algorithm and artificial NNS for music classification [9]. Cheng et al. developed and studied the first humming recognition system based on deep learning, which uses typical string matching-based recognition technology and uses the letters U, D, or S to characterize the pitch change of the audio signal to represent the humming audio signal using a string composed of these three characters, and then use the string matching algorithm to calculate the matching probability of songs in the database [10]. Zhang et al. applied the restricted Boltzmann machine to the classification of music genres and constructed a 5-layer restricted Boltzmann machine, but this method has an obvious defect that it can only be used in four. The accuracy rate of music genre classification is maintained above 50%. With the increase of the types of music genres classified, the classification accuracy rate will also decrease [11]. Li and Su concatenate Mel cepstral coefficients and perceptual properties such as fundamental frequency, spectral centroid, and sub-band energy to form high-dimensional feature vectors [12]. Li believes that computers, like people, are a physical symbol system, and the generation of intelligent behavior needs to be able to transform specific symbols or certain patterns of physics into other patterns and symbol systems [13]. The NNS developed by Xiongjun and Lv can imitate the human brain mechanism for data analysis. Its predecessor is the artificial NNS, and its basic feature is to try to imitate the pattern of information transmission and processing between neurons in the brain [14]. Ceylan et al. propose that affective computing is a computation that is related to emotions and originates from or can affect emotions. Traditional human-computer interaction cannot understand or adapt to human emotions or moods. This lack and limitation of the ability to understand and express emotions make it difficult to expect computers to have the same intelligence as humans in the future, and it is also difficult to see that human-computer interaction can be truly natural and harmonious in the future [15]. Humphrey et al. using AI technology presented the continuous analysis of learning results given by the system to teachers and students, including valuable reports on performance, students' learning status and learning attitude, and any mistakes made by students in the learning process and deviated understanding of the learning content [16]. Ferenc designed a computer system with intelligent algorithms based on AI. The system starts with minimal information, such as the type of instrument that plays the music, and then, without human intervention, it can create an extremely complex piece of music, often able to resonate emotionally with the audience within minutes [17]. Koempel argues that affective thinking also occurs in the neocortex, but is influenced by certain parts of the brain, including brain regions such as the amygdala, as well as some recently evolved brain structures such as spindle neurons, which appear to be involved in higher-level emotional aspects that play a key role [18].

The current issue is that excellent learning opportunities cannot be fairly provided to music learners who want to learn more deeply, whether they are zero-based piano students and parents or other music learners. The advancement of AI technology will end the limitations and impasses in this area and can offer music students excellent musical resources and equitable educational opportunities. The effectiveness and efficiency of music instruction will increase thanks to artificial intelligence technology. We can quickly and accurately understand students' learning process, learning background, personal strengths and weaknesses using big data analysis, artificial intelligence technology, and how it acts and reacts. More researchers are starting to look into how deep learning technology might be applied to the field of music information retrieval as a result of the excellent results that deep learning technology has produced in the fields of image recognition and speech recognition.

## 3. Theoretical Basis of Deep Learning

### 3.1. Backpropagation NNS

Deep learning has been developed from artificial NNSs, and research in artificial NNSs has started very early. The input of a neuron can come from both the input signal and the output of other neurons. A typical fully connected NNS has a large number of neurons and is divided into three layers: output layer, hidden layer, and input layer. The network structure has only one hidden layer, and the NNS is also called a single hidden layer feedforward NNS, as shown in Figure 1.

To enhance learning ability, multiple hidden layers can be set up in deep learning, and each hidden layer can have a different number of neurons depending on the situation. A NNS with various layers of neurons is connected. There is no connection between the neurons in the same layer; rather, the neurons of each layer are connected to the neurons of the layer before it. For the hidden layer and the output layer, each layer is multiplied by the connection weight matrix of the preceding layer, the output value of the neurons in the preceding layer, plus the bias term of the layer to obtain a linear output. Then, the layer is passed through the activation function. The output of the neurons in this layer is obtained through a nonlinear transformation [19]. The backpropagation algorithm can be thought of as a type of supervision learning algorithm because it determines the gradient of the loss function through the error term, and the error term is determined from the actual output value and the target output value through a specific mathematical rule. By applying the chain rule to iteratively compute the gradient of each layer, backpropagation generalizes the delta rule to a multi-layer feedforward NNS. Any supervised learning algorithm's objective is to identify the optimal function that converts a set of inputs into the desired output. The goal of the backpropagation algorithm is to train a multi-layer NNS so that it can develop a suitable internal representation that enables it to learn arbitrary input-to-output mappings. The process of neurons in each layer from receiving input to calculating output is shown as follows:

(1) $$\begin{array}{c} z^{l}=W^{l}a^{l}+x. \end{array}$$

Starting from the input layer, along the direction of input to output, according to the above process, the input vector, connection weight matrix, and bias term of each layer are subjected to a series of linear and activation operations, and then calculated layer by layer. Until the output layer obtains the target prediction result, such a process is a forward propagation process. Since the learning ability of multi-layer networks is much stronger than that of single-layer NNSs, more powerful learning algorithms are needed to train multi-layer networks [20]. Since the backpropagation algorithm is the most effective among many learning algorithms, the backpropagation algorithm is the most widely used learning algorithm for training NNSs.

A NNS that has just built its hierarchical structure does not yet have the ability to predict. It needs to be trained with training data so that the NNS can learn the predictive ability we expect. The learning process of the NNS is to iterate continuously according to the training data and adjust the connection weights and bias terms between neurons, so that the error of the final objective loss function calculation is minimized and the parameters are converged. The learning process of NNS includes forward propagation and backpropagation. An error occurs if the target predicted value is not equal to the expected output value. At this point, the process of the backpropagation algorithm is entered. According to the error loss function, the error of the output layer is calculated, and then it is reversely transmitted to the middle layers in some form, and the parameters of each layer are updated. By iterating continuously, the error of the loss function calculation is minimized and the parameters converge. The backpropagation algorithm uses gradient descent, as shown in the following equations:

(2) $$\begin{array}{c} w_{ij}^{l}=w_{ij}^{l}-\eta \Delta w_{ij}, \end{array}$$

(3) $$\begin{array}{c} x_{ij}^{l}=x_{ij}^{l}-\eta \Delta x_{ij}. \end{array}$$

The loss error is calculated according to the target prediction and expected output of the output layer as shown in the following equation:

(4) $$\begin{array}{c} L=\tau \left(a^{x},b^{M}\right). \end{array}$$

According to the error term, the connection weight of each layer and the gradient of the bias term are calculated as shown in the following equations:

(5) $$\begin{array}{c} \Delta x_{ij}^{l}=\frac{\partial L_{ij}^{l}}{\partial z}\cdot \frac{\partial z_{ij}^{l}}{\partial L}, \end{array}$$

(6) $$\begin{array}{c} \Delta w_{ij}^{l}=\frac{\partial L_{ij}^{l}}{\partial x}\cdot \frac{\partial x_{ij}^{l}}{\partial L}. \end{array}$$

The multi-layer is reflected in the sufficient number of deep NNS layers commonly used in deep learning, and the nonlinearity is reflected in the nonlinear transformation brought by the activation function to the network model. The activation function realizes delinearization, making the NNS a nonlinear model, and bringing the network model the ability to solve linear inseparable problems.

### 3.2. Bidirectional NNS Model

The layers of the NNS are no longer fully connected. A hidden unit can only connect a part of the input unit, and the corresponding image is that the hidden unit only connects a small adjacent area of the input image. The recursive use is that natural images have their inherent characteristics; that is, the statistical features of an image in a certain part are as applicable as the features of other parts [21]. In theory, the features extracted by recursion can be directly classified by traditional classifiers, but even the features after recursive processing still have a relatively high dimension, so generally a one-step downsampling process is performed after recursion. The output value of the bidirectional NNS is affected by the previous input values as shown in Figure 2.

In theory, a bidirectional NNS can look forward any number of steps. The training error cannot be propagated in more layers on the time axis. Similar to the forward network, the error at the earlier time point cannot be affected, and its weight cannot be updated, which will make the model difficult to train.

For model training in deep learning, a lot of training data is needed. The model effect improves with increased training data. Small data sets, however, are essentially unable to help the deep network model learn the knowledge it needs due to the model's complexity. Small data sets are insufficient for learning. Due to the high cost of labeling, many problems do not currently have enough labeled training data sets. As a result, deep network models cannot be used to solve these small data set problems, and only some conventional models can. The human brain served as inspiration for the NNS proposal. The earliest and most basic network model is the neuron, but the initial NNS was unable to resolve the XOR issue. The NNS model has culminated. Deep learning is currently excelling in a number of fields, particularly the field of images. It has consistently shattered earlier historical records and is currently the hottest cutting-edge technology.

## 4. Intelligent Music Classification Based on Deep Learning

### 4.1. Classification of Music Teaching Genres

The rapid advancement and development of modern scientific and technological means have had a significant negative impact on music education, posing significant challenges and requiring material and technical changes. Innovation plays a crucial role in advancing development, which cannot be understated. Positive changes and influences have been brought about as a result of the development of various modern music education theories, new ideas, and improved teaching techniques. Electronic musical instruments have become increasingly intelligent and humanized as AI technology continues to advance. In addition to storing more musical instrument timbres, this type of intelligent musical instrument can also arrange various timbres. In accordance with specific behavioral instructions, various timbres are played in succession. This musical instrument performs in a way that is unmatched by previous musical instruments. This situation offers a fresh approach to teaching music education. Assembling various musical instruments to create something together while using their own ideas allows students to better practice their musical skills in the classroom, which enhances the effectiveness of music instruction. Due to the significant advancements in the quality and arrangement of the music produced by these instruments, a new music function has taken the place of the original manual mode, and numerous intelligent and humanized music programming functions have replaced the previous clumsy operation mode. Consequently, music education has widely promoted the use of these instruments. The use of such musical instruments has increased, whether it be in music education at universities or in primary and secondary schools. Music education becomes more standardized with an accurate scoring system. A score example will appear on the split screen of the student side when students practice and play music using the intelligent system, and they will begin to play along with the accompaniment. When the notes are played properly, the notes on the screen will also play back properly. If you play the incorrect note, the screen will show you what it is and mark the incorrect time, whether it is a rush or a drag, making the student's error immediately obvious. As part of a multi-classification task, the categories used in this section's experiments to classify music genres for intelligent music teaching of various music genres are fairly evenly distributed.

AI technology can quickly stratify complex large-scale music or sections, simplify teaching, make it easier for students to understand music, effectively solve students' difficult problems in class, simplify the tasks of teachers, and effectively pull in the course. The distance between the teacher and the recipient has been shortened, the traditional music education model has been changed, and the bold innovation of the music education model has been realized. In music enlightenment education, intelligent music teaching has made great progress. For music enlightenment education, intelligent music teaching should pay more attention to the positive interaction between students and intelligence, and let students start from music itself and fall in love with this art form, not just by simply playing games to arouse students' interest. AI equipment can help music learners to practice and perform more conveniently, whether it is an intelligent electro-acoustic musical instrument or an intelligent teaching system, etc., all for music learners to achieve better results in their practice and performance. I believe that in the near future, AI can solve more problems we encounter in the practice process, and can also provide assistance for better performances. Music genre classification is an important branch of music information retrieval. Correct music classification is of great significance to improve the efficiency of music information retrieval.

The approach used in this paper can be broken down into two parts for the purpose of identifying the various musical genres. The first step is feature engineering, also known as feature extraction. Mel cepstral coefficients, spectral centroid, and spectral contrast are the three features that this paper will extract as they can best represent audio content. The extracted features will then be input into the neural network we have designed in this paper for training, and we will output the classification result at the end. This paper firstly inputs the Mel cepstral coefficient, spectral centroid, and spectral contrast into the NNS as a single feature, observes the experimental results, and then fuses the features in pairs. Finally, the Mel reversed to determine the best method; the spectral coefficient, spectral centroid, and spectral features are all input into the NNS simultaneously. The results are then compared to the results of a single feature. In this study, the data set is divided into three portions at random and used as the training set, validation set, and test set, respectively. The proportion of the three data sets is shown in Figure 3.

### 4.2. Data Set Classification Processing Simulation

Correct music genre classification not only helps to improve the efficiency of music teaching, but also helps to improve the accuracy of music recommendation. The characteristic of music teaching data is to select only the spectral contrast. Because the spectral centroid contains too little data information, it is not suitable to be input into the NNS as a single feature as a comparison experiment, and it is suitable to be used as the enhanced data of the NNS and the spectral contrast. The features selected for each experiment are shown in Table 1.

The experimental parameters of this feature set are shown in Table 2.

Since the spectral contrast of the neural network model and the spectral centroid are among the features extracted by the data preprocessing part, their minimum and maximum dimensions are 12 and 36, respectively. As a result, the input layer's number of neurons will fluctuate between 12–36 depending on the feature combinations used. The context information between the features is extracted from the hidden layer, and the hidden layer's current state is used to calculate the output state at the moment. The input of the network is extracted, and the parameter matrix is initialized using the gliffy uniform distribution initialization method. The output is the classification probability for each genre, and the input is a feature vector for the time series.

### 4.3. Analysis of Experimental Results

The entire experimental process is mainly a comparative experiment. The experimental music data feature only selects the music teaching genre NNS model, and the data feature only selects the spectral contrast. Because the spectral centroid contains too little data information, it is not suitable for input into the LSTM network as a single feature. As a comparative experiment, it is suitable to be used as enhanced data for NNSs and spectral contrast. In this paper, the spectral centroid is used as a separate feature to conduct an experiment and the three features of spectral contrast are fused and input into the NNS. The experimental results are shown in Figures 4–6.

It can be seen from Figure 6 that the accuracy of feature 1 and feature 3 on the training set is very high, but the accuracy on the test set is very low, which indicates that the model is overfitting and the generalization ability of the model is too poor. From the feature data selected by feature 1 and feature 3, it can be analyzed that the neural network model was selected in both experiments, which also shows that neural network is indeed the most important feature in speech signal processing, and it is the most effective way to describe audio content. Characteristics: In this paper, it is found that the classification accuracy of using spectral contrast alone is higher than that of spectral contrast and spectral centroid fusion. Classification effect: Because the features can influence each other, how to combine the features to achieve the best classification effect requires continuous experimentation. Select feature 1 and feature 3 models for error experiments, as shown in Figures 7 and 8.

The short-time Fourier spectrogram and Mel spectrogram of the music must be extracted as input data for the deep learning method in order for the NNS to automatically learn the abstract spectrogram features. This study also manually extracts several features from the audio data in order to compare it to the conventional machine learning classification method. The extracted feature data are then fed into the model with the conventional machine learning classification method acting as the classifier for training. This study, which uses experimental analysis to support its findings, demonstrates that different music teaching genres can be accurately classified at a rate of over 90%, which has a positive impact on recognition. The NNS model put forth in this paper can make it easier for music students to practice and perform, whether it be with an intelligent electric-acoustic instrument or an intelligent teaching system, etc., all of which are aimed at helping students of music to improve their practice and performance. I think artificial intelligence will soon be able to assist us in improving our performances and solve more of the issues we face during practice. Students will become more active in the classroom this way, moving from being passive.

## 5. Conclusions

The use of AI in our studies and daily lives has increased, and this trend has also been seen in the teaching of music. Particularly, the extensive application of AI in modern music education not only dismantles the traditional music education model, but also offers schools a new music teaching model suitable for students to learn, so that students can better learn music knowledge in the process of learning music, to gain a deeper understanding of the characteristics and functions of each musical character and element. It not only enhances the relationship between teachers and students in music education, but also gives students the opportunity to become more integrated into the larger music community, continuously learn new music, enjoy music, and make music. AI technology has the ability to quickly stratify complex large-scale music or sections, simplify instruction, improve student understanding of music, efficiently solve challenging student problems in class, make tasks for teachers simpler, and efficiently pull in the course. The bold innovation of the music education model has been realized, and the distance between the teacher and the student has been reduced. In order to classify music based on its content, features are typically manually extracted and then entered as training data into a model using conventional machine learning classifiers. There are two main components to later researchers' primary work. On the one hand, the task is to identify the characteristics that can accurately describe the musical content. On the other hand, the work mainly focuses on enhancing the classifier's algorithm. The classification accuracy rate of the various music teaching genres in this paper reaches more than 90%, which has a good recognition effect, as shown by experimental analysis. Whether it be an intelligent electric-acoustic musical instrument, an intelligent teaching system, etc., the NNS model put forth in this paper can assist music students in practicing and performing more conveniently. I think artificial intelligence will soon be able to help us with more practice-related issues and improve our performances. The accuracy of the neural network model in classifying musical genres is found in this paper to be the highest among the methods used, but other neural network structures can still be tested. For instance, the output of the convolutional neural network can be used as the input of the cyclic neural network.

## Figures and Tables

**Figure 1:** NNS structure diagram.

**Figure 2:** Bidirectional NNS model.

**Figure 3:** The proportion of the data set.

**Figure 4:** Comparison of the accuracy of the feature one model.

**Figure 5:** Comparison of the accuracy of the feature two models.

**Figure 6:** Accuracy comparison of feature three models.

**Figure 7:** Feature model error comparison.

**Figure 8:** Error comparison of three feature models.

**Table 1:** Correspondence of experimental feature selection.

Experimental feature set	Feature selection
1	NNS collection
2	Spectral contrast
3	NNS + spectral centroid
4	Spectral contrast + spectral centroid
5	NNS + spectral contrast

**Table 2:** Experimental parameters.

Experimental parameters	Value
Learning rate	0.005
Batch size	50
Rounds	300
Dropout	0.07
Activation function	Softmax
Optimizer	categorical_crossentropy
Loss function	Adam

## Data Availability

The data used to support the findings of this study are included within the article.
